# Pseudopodium enriched atypical kinase 1(PEAK1) promotes invasion and of melanoma cells by activating JAK/STAT3 signals

**DOI:** 10.1080/21655979.2021.1961661

**Published:** 2021-08-09

**Authors:** Min Pan, Xiaohui Yin, Yi-chuan Huang

**Affiliations:** a Department of Dermatology, The Affiliated Hospital of Qingdao University, Qingdao, China; b Department of Dermatology, Qingdao Women and Children’s Hospital, Qingdao, China; c Department of Otolaryngology, The Affiliated Hospital of Qingdao University, Qingdao, China

**Keywords:** Melanoma, metastasis, pseudopodium enriched atypical kinase, JAK/STAT3 signals

## Abstract

Pseudopodium enriched atypical kinase 1(PEAK1) is a non-receptor tyrosine kinase, which is enriched in the pseudopodia of migrating cells and plays an important role in regulating cell migration and proliferation. In the study, we investigate the therapeutic effect of PEAK1 on melanoma cells *in vitro* and *in vivo*. We used a lentiviral vector to express short hairpin RNAs (Lv-PEAK1 shRNA) for inhibiting PEAK1 expression in the melanoma SKMEL28 cells. A full-length PEAK1 gene was cloned into the pcDNA 3.1 (+) plasmid and used to infect the melanoma SKMEL19 cells. P6 (also known as Pyridines 6, EMD Chemicals), the Pan-JAK inhibitor, was used to inhibit the Janus kinase/signal transducer and activator of transcription 3 (JAK/STAT3) pathway. The cell counting kit-8 (CCK-8), colony formation assay and transwell assay were used to detect cell proliferation, growth and invasion *in vitro*. The effect of PEAK1 on melanoma progression *in vivo* was also evaluated. Protein expression of PEAK1, E-cadherin, vimentin and JAK/STAT3 was measured using western blot assay or immunohistochemistry. The results showed that enforced PEAK1 expression facilitated melanoma cell growth, invasion and metastasis via activating JAK/STAT3 signals, and PEAK1 knockdown inhibited melanoma cell growth, invasion and metastasis via inactivating JAK/STAT3 signals. Further work demonstrated that P6 (500 nM) treatment reversed PEAK1-induced effect in melanoma cells. PEAK1 promotes tumorigenesis and metastasis via activating JAK/STAT3 signals, and PEAK1 knockdown reduced tumorigenesis and metastasis in melanoma via inactivating JAK/STAT3 signals, providing a novel therapeutic strategy for melanoma treatment.

## Introduction

Melanoma is the most deadly malignancy of the skin, which frequently metastasizes to distant organs such as bone, lung, liver and brain [1,2]. Melanoma is nearly resistant to all clinical therapy with a median survival time of only 6–9 months and a 3-year survival of 15% [3–6]. Therefore, it is very important to clarify the molecular mechanism of metastasis and could launch clinical-translational initiatives in patients with melanoma [6].

The activation abnormalities in the signal transducer and activator of transcription 3 (STAT3) signaling pathway are associated with tumor onset and progression [7,8]. The activation of this pathway is regulated and controlled by the upstream factor Janus kinase (JAK). The JAK/STAT3 pathway played a crucial role in regulating cell proliferation and inflammation [8]. Persistent JAK/STAT3 signal transduction plays a crucial role in tumorigenesis and immune development. JAK2/STAT3 activation promotes cell metastasis and increases cell motility via induction of epithelial–mesenchymal transition (EMT) and activation of focal adhesion kinase (FAK) [9]. The JAK/STAT pathway is also essential for many developmental processes including cellular proliferation, innate immune responses, stem cell differentiation and maintenance. In colorectal cancer (CRC) HCT116 and HT29 cells, TGF-β1 induces differentiation of MSCs into CAFs and promotes the migration and invasion of HCT116 and HT29 cells via activating JAK/STAT3 signaling pathway, which ultimately accelerates the formation of TME for liver metastasis [10]. Activated JAK/STAT3 signaling has been validated as a promising molecular target for cancer therapeutics discovery and development. In human melanoma cells, the pan-JAK inhibitor 6BIO can effectively induce tumor cell apoptosis by inhibiting JAK/STAT3 signaling [11].

Pseudopodium-enriched atypical kinase 1 (PEAK1) is a non-receptor atypical tyrosine kinase family member sgk269, which contains an N-terminal actin-targeting region and a functional C-terminal atypical kinase domain [12]. The domain structure of PEAK1 has predicted consensus binding and/or substrate sites for Src, Erk, Shc and Crk and can operate within Src-p130Cas-Crk-Paxillin and Ras-Raf-Erk signaling pathways to regulate cell proliferation, migration and cancer progression [12,13]. In addition, PEAK1 is ubiquitously expressed in multiple tissues, suggesting that it has a major role in normal physiology by regulating these signals. Research has been reported that PEAK1 plays a positive role in regulating cell growth, invasion and metastasis in human lung cancer [14], colorectal cancer [15], breast cancer [16] pancreatic ductal adenocarcinoma [17] and therapy resistance in human pancreatic ductal adenocarcinoma [18]. In addition, PEAK1 mediates TGF-β signaling and controls extracellular microenvironment in tumor cells [19]. In breast cancer cells, PEAK1 mediates TGF-β receptor signals and integrin/Src/MAPK pathways and regulates TGF-β-induced epithelial–mesenchymal transition (EMT) and metastasis [15]. In lung cancer cells, enforced PEAK1 expression induces EMT via activating extracellular signal-regulated kinase-1/2 (ERK1/2) and Janus kinase-2 (JAK2) signaling [9]. In PDAC or cells, increased expression of PEAK1 occurs in PDAC, and overexpression of PEAK1 in pancreatic ductal epithelial cells promotes acquisition of a migratory and invasive phenotype through enhanced JAK/STAT signaling [17]. However, the role and mechanisms of PEAK1 in melanoma invasion is still unknown.

Since PEAK1 has the ability to induce EMT and promote cancer cell metastasis, it is speculated that PEAK1 has a similar effect on melanoma cells. In the study, we aimed to determine the role and mechanisms of PEAK1 in regulating cell invasion and metastasis in melanoma cells *in vitro* and *in vivo*. We found that enforced PEAK1 expression promotes cell growth, invasion and EMT-related traits via activating JAK/STAT3 signaling, and PEAK1 knockdown inhibits cell growth, invasion and EMT-related traits via inactivating JAK/STAT3 signaling. We also found that targeting JAK/STAT3 signaling reversed PEAK1-induced effects, which provided a novel therapeutic target for melanoma.

## Materials and methods

### Cell culture

Melanoma cell lines SKMEL-1, SKMEL-2, SKMEL-19 and SKMEL-28 were obtained from the American Type Culture Collection (ATCC; Shanghai, China). They were cultured in Dulbecco’s modified Eagle’s medium supplemented with 10% FBS at 37°C.

### shRNA transfection and lentivirus production

PEAK1 shRNA-pLKO.1 constructs were obtained from Open Biosystems (Huntsville, AL). Four shRNAs were used for PEAK1 knockdown, and only one shRNA sequence with 90% efficiency to target PEAK1 was used for further experiments. The PEAK1 targeted sequences used for further experiments are 5ʹ-ATAGGGAGGGTGGGATCAGTCTTGAGGAC-3; control/Scramble: 5ʹ-GGCATTACAGTATCGATCAGA-3ʹ. 293 T cells (1 × 10^6^) were plated in a 35 mm dishes, and transduced approximately 8 hr later with 2 µg total of the PEAK1 shRNA-pLKO.1 constructs. Lentivirus preparations were produced with a standard third-generation packaging system. Viral supernatants were supplemented with 8 μg/mL polybrene and incubated with cells for 48 h. SKMEL28 cells were harvested 1 to 5 days and selected with 1 µg/mL puromycin for stable colonies (Lv-PEAK1 shRNA and Lv-NC).

### Plasmids and transfection

A full-length PEAK1 gene was cloned into pcDNA 3.1 (+) plasmid (PEAK1) which used to increase PEAK1 overexpression in the cells, and pcDNA 3.1 (+) (NC) plasmid was as the control. The pcDNA3.1 (+)-PEAK1 (PEAK1) and control pcDNA3.1 (+) (NC) plasmid were amplified and purified and transfected into SKMEL19 cells using Lipofectamine 3000 (ThermoFisher Sci) as the manufacturer’s protocol. After 48 h transfection, the cells were selected using 1 µg/ml puromycin for 1 week. In addition, cells transiently transfected with pcDNA3.1 (+)-PEAK1 (PEAK1) or pcDNA3.1 (+) (NC) for 1–5 days was used for further analyses. All plasmids were sequenced to ensure the orientation and correct reading frame. The stable colonies were named pcDNA3.1 (+)-PEAK1 (PEAK1) and pcDNA3.1 (+) (NC).

### CCK-8 assay

Cells (1 × 10^4^/well) were transfected with PEAK1 (SKMEL19) or PEAK1 shRNA (SKMEL28) or their control for 24–120 h. To explore the effect of PEAK1 on JAK/STAT3 signal, SKMEL19 cells were treated with P6 (500 nM) [Calbiochem (Nottingham, UK)] or control DMSO for 8 h, then transiently transfected with PEAK1 or PEAK1 shRNA for 24–120 h. The cell proliferation was detected using CCK-8 assay kit (Dojindo, Kumamoto, Japan) as the manufacture’s instruction.

### Colony formation assay

The stable Lv-PEAK1 shRNA transfected SKMEL28 cells or the stable PEAK1 transfected SKMEL19 cells or their controls (1 × 10^3^) were seeded into 6-well plates and cultured for 10 days. To explore the effect of P6 on colony formation, the stable PEAK1 transfected SKMEL19 cells were seeded (1 × 10^3^) in six well plates and treated with vehicle (DMSO) or P6 (500 nM) for 3 days. Fresh media without P6 was then added to the cells and cultured for another 7 days. After which, the cells were fixed and stained with May-Grunwald-Giemsa. The number of colonies was counted and reported in graphs.

### Cell migration and invasion assays

Lv-PEAK1 shRNA or Lv-NC transfected SKMEL28 cells, PEAK1 or NC transfected SKMEL19 cells or PEAK1/P6 (500 nM) treated SKMEL19 cells were seeded at the density of 1 × 10^5^ cells/100-mm culture plate for 24 h in transwell inserts pre-coated by Matrigel (BD Biosciences, Hangzhou China) as previously reported [20]. The migration assays were performed similarly to the invasion assays, except the inserts were not conducted with pre-coating of Matrigel. The membrane was photographed from five fields at a 200× magnification and the number of cells was counted. All experiments were repeated three times.

### Wound healing assay

Lv-PEAK1 shRNA or Lv-NC transfected SKMEL28 cells, PEAK1 or NC transfected SKMEL19 cells were grown to confluence and treated as indicated. To explore the effect of P6 on colony formation, the SKMEL19 cells were treated with P6 (500 nM) for 48 h, then transfected with PEAK1 or NC. After 24 h, a wound was made in the monolayer with a sterile pipette tip, the cells were washed to remove debris and new low-serum medium (containing 0.5% FBS) was added. Phase-contrast images of the wounded area were captured at 0 and 72 h after wounding using the 10X objective of a Zeiss Observer Z1 microscope operated by the Zen software (Zeiss, Oberkochen, Germany). Wound widths were measured at 11 different points for each wound, and the average rate of wound closure was calculated (in μm/hr) using the ImageJ software.

### Western blot assay

Cells were collected and the extracts were prepared in RIPA buffer (Cell Signaling Technology, Shanghai, China) supplemented with Complete protease inhibitor cocktail (Roche) at 4℃ for 40 min and then separated by electrophoresis, incubated with anti-PEAK1, anti-E-cadherin, anti-vimentin, anti-JAK1/2, anti-phospho-JAK1/2, anti-STAT3, anti-phospho STAT3 (Cell Signaling Technology), β-actin (Abcam, Cambridge, UK) antibodies. The western blots were representative of n = 3.

### *In vivo* studies

The studies *in vivo* were conducted and approved by the Institutional Animal Care and Use Committee of the affiliated hospital of Qingdao University. The experiments were divided into four groups as below: ① PEAK1 shRNA/SKMEL28 cells ② NC shRNA/SKMEL28 cells ③ PEAK1/SKMEL19 cells ④ NC/SKMEL19 cells. 5 × 10^6^ cells/0.1 ml PBS were subcutaneously or intravenously through the tail vein injected into the flanks of 5-week-old nude mice (n = 5/group). Tumor volumes were measured at 5-day intervals and calculated as length × width^2^ × 0.4. The tumor masses were excised and the lungs were removed for further analysis.

### Immunohistochemistry

Tissue sections (5 μm) of tumor xenograft or metastatic lung nodes were deparaffinized and blocked and incubated with primary antibody (Cell Signaling, Shanghai, China) against PEAK1 and Ki67 (tumor xenograft), E-cadherin and vimentin (metastatic lung nodes). Then, the slides were incubated with HRP-conjugated secondary antibody and peroxidase activity was visualized using a substrate solution of diaminobenzidine (DAB) containing 0.03% hydrogen peroxid, and counterstained with Harris hematoxylin. Tissue sections were washed in water, dehydrated, cleared, mounted and observed using Olympus FLUOVIEW Viewer software (Tokyo, Japan). Within the tissue core, the most representative tumor area of standardized size was selected at ×200 magnification. The staining intensity in this area was measured if the area contained >5% epithelial cells. Stains were scored as negative (−), weak (+), intermediate (++), and strongly positive (+++) as reported [14].

### Statistical analysis

For all assays and analyses *in vitro*, if not specified, student’s t-test was used to evaluate the significant difference or p-values and standard deviations (SD) of mean values were depicted as error bars in figures. For animal studies *in vivo*, Shapiro–Wilk test was applied to check the normality of the raw data, and student’s t-test was applied in exploring the P-value and the significant differences between groups. Data analyses were performed t-test in SPSS22.0 soft. Statistical significance was determined by *p < 0.05. **p < 0.01, ***p < 0.001.

## Results

### Enforced PEAK1 expression promoted cell migration and invasion *in vitro*

PEAK1 expression was detected in melanoma cell lines (SKMEL-1, SKMEL-2, SKMEL-19, SKMEL-28) by western blot assay. As shown in Figure 1(a), highest PEAK1 expression was found in the SKMEL-28 cells, and lowest PEAK1 expression was found in SKMEL-19 cells. So, we used SKMEL-28 and SKMEL-19 cells for further study.

**Figure 1.** PEAK1 plays a critical role in migration and invasion in melanoma cells in vitro

A, PEAK1 protein expression was detected by western blot assay in SKMEL-1, SKMEL-2, SKMEL-19 and SKMEL-28 cells. B, PEAK1 protein was detected by western blot assay in SKMEL-19 cells transfected with PEAK1 or control for 48 h. C, PEAK1 protein was detected by western blot assay in SKMEL-28 cells transfected with PEAK1 shRNA or control NC shRNA for 48 h. D, E, transwell migration assay and transwell invasion assay in PEAK1 or control transfected SKMEL-19 cells. F, G, transwell migration and invasion assay in PEAK1 shRNA or control NC shRNA transfected SKMEL-28 cells.

pcDNA3.1-PEAK1 (PEAK1) and pcDNA3.1 (NC) was transiently transfected into the SKMEL19 cells for 24 h. The transfection efficiency was confirmed by western blotting. PEAK1 expression was increased in the PEAK1-transfected SKMEL19 cells compared to the NC transfected SKMEL19 cells (Figure 1(b)). PEAK1 shRNA and NC shRNA were transiently transfected into the SKMEL-28 cells for 24 h. PEAK1 expression was decreased in the PEAK1-transfected SKMEL-28 cells compared to the NC shRNA transfected SKMEL-28 cells (Figure 1(c)).

PEAK1 was reported to be overexpressed in the human multiple cancer tissues than the normal tissues, and higher PEAK1 expression is associated with poor disease prognosis. In colorectal cancer cells, silencing PEAK1 inhibits cell proliferation, migration, and invasion *in vitro* and inhibits the growth of tumor xenografts in nude mice [12]. We next focused on whether PEAK1 gene silencing or overexpression influences the migration and invasion ability of SKMEL19/28 cells *in vitro*. The results showed that over-expression of PEAK1 protein could significantly promote the migration (Figure 1(d)) and invasion (Figure 1(e)) of SKMEL-19 cells, while decreasing PEAK1 protein could significantly decrease cell migration (Figure 1(f)) and invasion (Figure 1(g)) of SKMEL-28. Wound-healing assays also showed that PEAK1 shRNA inhibited cell migration and PEAK1 promoted cell migration (Figure 2).

**Figure 2.** PEAK1 regulates SKMEL19/28 cells migration *in vitro* by wound healing assay

SKMEL19 cells were transfected with PEAK1 or NC, SKMEL28 cells were transfected with PEAK1 shRNA or NC shRNA. Cells were then grown in a monolayer, wounded and left to recover the wound then imaged at the same frame after 48 h. The graph is a quantitation of the wounds. Wound widths were measured at 11 different points for each condition and the average rate of wound closure was calculated in μm/hr. Data are the mean −/+ SEM from 3 wound closure assays and *p < 0.01. Scale bar is 200 μm.

EMT is a development program that initiates metastatic dissemination of cancer cells from the primary tumor, and promotes mesenchymal phenotypes with increased migratory and invasive capabilities [21]. It is a complex process that can inhibit cell–cell connections and apicobasolateral polarity in epithelial cells, with decreased expression of epithelial markers (such as E-cadherin and β-catenin) and increased expression of mesenchymal markers (such as vimentin and N-cadherin) [22]. PEAK1 overexpression has shown to induce epithelial-to-mesenchymal transition (EMT) *in vitro* and *in vivo*, whereas PEAK1 knockout had the opposite effects [14]. To determine whether PEAK1 can promote EMT of SKMEL-19 cells and targeting PEAK1 can inhibit EMT of SKMEL-28 cells, we examined the E-cadherin and vimentin levels in the PEAK1 overexpressing SKMEL-19 cells and the PEAK1 downexpressing SKMEL-28 cells. As shown in Figure 3(a), the E-cadherin protein level was down-regulated and the vimentin levels were up-regulated in the SKMEL-19 cells with PEAK1 overexpression. On the contrary, the E-cadherin protein level was up-regulated and the vimentin levels were down-regulated in the SKMEL-28 cells with PEAK1 knockdown (Figure 3(b)), suggesting that PEAK1 regulated cell invasion through EMT.

**Figure 3.** PEAK1- induced cell invasion and migration by regulating JAK/STAT3 signals

A, JAK/STAT3 signals were detected in NC or PEAK1 transfected SKMEL-19 cells by western blot assay. B, JAK/STAT3 signals were detected in NC shRNA or PEAK1 shRNA transfected SKMEL-28 cells by western blot assay. C, SKMEL-19 cells were treated with P6, then transfected with NC or PEAK1 for 48 h, cell invasion was detected by transwell invasion assay. D, SKMEL-19 cells were treated with P6, then transfected with NC or PEAK1 for 48 h, cell invasion was detected by transwell migration assay.

### Effect of PEAK1 on the JAK/STAT3 signals

We next evaluated whether PEAK1 observed in these models was associated with activation of the JAK/STAT3 pathway. In the present study, we found that enforced PEAK1 expression promoted JAK1/2 phosphorylation and STAT3 phosphorylation (Figure 3(a)). In contrast, targeting PEAK1 significantly reduced JAK1/2 phosphorylation and STAT3 phosphorylation (Figure 3(b)).

### Targeting JAK/STAT3 attenuated PEAK1-induced EMT and cell invasion

JAK/STAT3 signaling, which regulates many aspects of cancer development and progression, promotes invasion and metastasis through activation of key metastasis promoting genes [23]. Increased expression of SgK223, a pseudokinase and scaffolding protein closely related to PEAK1 promotes acquisition of a migratory and invasive phenotype through enhanced JAK/STAT3 signaling in pancreatic ductal epithelial cells [17]. Next, we tested whether inhibiting JAK/STAT3 pathways could reduce invasion caused by PEAK1. To do this, we used the stable PEAK1 transfected SKMEL19 cells in invasion and migration assays. Cells were incubated with 500 nM P6. In the PEAK1-overexpressing SKMEL19 cells, P6 inhibited PEAK1-mediated JAK/STAT3 signaling after 24 h of treatment (Figure 3(a)). In addition, cell proliferation was obviously decreased with P6 treatment in the PEAK1 overexpressing cells (data not shown). Knockdown of JAK/STAT3 pathways partially reversed the promoting effect of PEAK1 on cell invasion (Figure 3(c)) and migration (Figure 3(d)) *in vitro*, suggesting that JAK/STAT3 pathway was involved in PEAK1-mediated cell invasion and migration. JAK-STAT3 activation has been reported to regulate the expression of a variety of important genes. Further analysis demonstrated that targeting JAK/STAT3 signal partially rescued the expression of E-cadherin and vimentin induced by PEAK1 overexpression (Figure 3(a)). Collectively, the data above strongly indicated that JAK/STAT3 -mediated EMT was regulated by PEAK1.

### PEAK1 promoted metastasis *in vivo*

Enhanced PEAK1 expression has reported to promote metastasis and tumor growth in pancreatic cancer [24], breast Cancer [15], lung cancer [9] and colorectal cancer [14]. We next investigated the role of PEAK1 in mediating SKMEL-19/28 cell metastasis in the mouse model. We first successfully achieved four types of modified SKMEL-19/28 cell lines: SKMEL-19 cells stably transfected with infected with control pCDNA3.1 (+) (NC) and pCDNA3.1 (+)-PEAK1 (PEAK1); SKMEL-19 cells stably transfected with Lv-PEAK1 or Lv-NC shRNA. Subsequently, we injected these four modified cell lines into female nude mice (5 weeks, 22–24 g) through the tail vein. By *in vivo* metastatic melanoma models, we found that enforced PEAK1 expression markedly increased lung metastatic nodes in the SKMEL19 cells, whereas targeting PEAK1 abrogated lung metastasis of SKMEL28 cells (Figure 4(a-b)), and few tumor masses could be seen in the lungs, suggesting that PEAK1 plays critical roles in melanoma cell metastasis.

**Figure 4.** PEAK1 plays a critical role in lung metastasis in melanoma cells in vivo

A, SKMEL19/PEAK1 or NC cells were i.v tail vein injected into nude mice for 35 days. Lung metastatic nodes were counted in the lungs. B, SKMEL28 /Lv-NC shRNA or Lv-PEAK1 shRNA cells were i.v tail vein injected into nude mice for 35 days. Lung metastatic nodes were counted in the lungs. C, E-cadherin expression was detected in metastatic lung nodes of PEAK1 or NC transfected mices. D, E-cadherin expression was detected in metastatic lung nodes of Lv-NC shRNA or Lv-PEAK1 shRNA transfected mices. E, vimentin expression was detected in metastatic lung nodes of PEAK1 or NC transfected mices. F, vimentin expression was detected in metastatic lung nodes of Lv-NC shRNA or Lv-PEAK1 shRNA transfected mice.

Mouse lung tissues were also sectioned for immunohistochemical staining for detecting E-cadherin and vimentin expression. The results showed that lung tumors with PEAK1 overexpression had lower levels of E-cadherin (Figure 4(c)) and higher levels of vimentin (Figure 4(e)) expression. On the contrary, lung tumors with PEAK1 down-expression had higher levels of E-cadherin (Figure 4(d)) and lower levels of vimentin (Figure 4(f)) expression.

### PEAK1 promoted cell proliferation *in vitro* and tumor growth *in vivo*

Colony formation and CCK-8 assay were employed to examine the effects of PEAK1 on SKMEL-19/28 cell growth. The results showed that colony formation ability was significantly promoted by PEAK1 over-expression in SKMEL-19 cells (Figure 5(a)) and significantly decreased in SKMEL-28 cells with PEAK1 knockdown (Figure 5(b)). CCK-8 assay showed that the enforced PEAK1 increased cell proliferation index in SKMEL19 cells (Figure 5(c)) *in vitro*, whereas knockdown of PEAK1 decreased cell proliferation index in SKMEL28 cells (Figure 5(d)) *in vitro*.

**Figure 5.** PEAK1 plays a critical role in melanoma cell growth *in vitro* and *in vivo.*

Cell growth was detected by colony formation assay in SKMEL19/PEAK1 or NC cells (A) and SKMEL28/Lv-NC shRNA or Lv-PEAK1 shRNA cells (B). Cell proliferation assay by CCK-8 assay in SKMEL19/PEAK1 or NC cells (C) and SKMEL28/Lv-NC shRNA or Lv-PEAK1 shRNA cells (D). SKMEL-19/PEAK1 or NC (E) or SKMEL28/Lv-NC shRNA or Lv-PEAK1 shRNA cells (F) were inoculated subcutaneously into nude mice. Xenografts were measured every 5 days with a caliper. PEAK1 (G) and Ki-67 (H) expression was detected in SKMEL19 Xenografts. PEAK1 (I) and Ki-67 (J) expression was detected in SKMEL28 Xenografts.

*In vivo*, enforced PEAK1 expression promoted growth of subcutaneous tumor cells (Figure 5(e)), and targeting PEAK1 expression suppressed growth of subcutaneous tumor cells (Figure 5(f)). Cell proliferation *in vitro* was assessed by Ki-67 staining. The results showed that PEAK1 was overexpressed in the SKMEL-19 tumor (Figure 5(g)), and PEAK1 was downexpressed in the SKMEL-28 tumor (Figure 5(h)). Enforced PEAK1 expression increased Ki-67 index (Figure 5(i)), and PEAK1 overexpression increased Ki-67 index (Figure 5(j)), indicating the oncogenic role of PEAK1 on melanoma.

## Discussion

This study indicated that enforced PEAK1 expression promotes cell proliferation, migration and invasion, and induces epithelial–mesenchymal transition (EMT) *in vitro*. Enforced PEAK1 expression activated JAK/STAT3 signal pathway, and enhanced the expression of vimentin and decreased the expression of E-cadherin. Furthermore, enforced PEAK1 expression promoted tumor growth and metastasis and EMT *in vivo*, and vice versa *in vitro*.

Previous studies have identified PEAK1 as a positive regulator of cell growth and metastasis in lung cancer [9], breast cancer [15] and pancreatic cancer [24]. However, the role of PEAK1 in melanoma remains unknown. Here, we found that downregulation of PEAK1 inhibited melanoma cell invasion, migration, and proliferation, and enforced PEAK1 expression promoted melanoma cell invasion, migration, and proliferation. We then investigated possible pathways by which PEAK1 could be involved in melanoma. Our studies showed that down-regulating PEAK1 inactivated JAK/STAT3 signaling. Recently, numbers of studies have shown roles for activated JAK/STAT3 signaling in the regulation of metastasis and proliferation in cancers. The above studies suggest that downregulation of PEAK1 expression decreases JAK/STAT3 signaling, thereby decreasing melanoma cell invasion, migration, and proliferation. On the contrary, PEAK1 overexpression promotes JAK/STAT3 signaling, thereby increasing melanoma cell invasion, migration, and proliferation.

EMT acts as a key regulator of metastasis by facilitating cancer cell invasion and distant dissemination [25,26]. During EMT, the transcription factors of EMT and matrix metalloproteases are upregulated to maintain a mesenchymal/invasive phenotype [27,28]. Several transcription factors, such as Twist, Snail, and Slug, have been reported to be involved in EMT via repressing specific epithelial cell marker E-cadherin and promoting specific mesenchymal cell marker vimentin and N‐cadherin [25,29]. In the present study, enforced PEAK1 inhibited E-cadherin expression, and promoted vimentin expression and PEAK1 knockdown promoted E-cadherin expression, and reduced vimentin expression in melanoma cells, suggesting that PEAK1 is associated with invasion and metastasis through regulating EMT.

It has been reported that targeting STAT3 affected cell proliferation and migration in cancer cells [30,31], and activation of JAK/STAT3 signaling pathway via enhancing EMT increases tumorigenic and metastatic ability and chemoresistance in cancer cells [32]. JAK/STAT3 signaling could be activated by cytokines [33], growth factors [34], intracellular proteins [35], including non-receptor kinases [36,37]. In the study, enforced PEAK1 expression promoted JAK1/2 and STAT3 phosphorylation, whereas PEAK1 knockdown has the contrary effect. In addition, PEAK1-induced effect in melanoma cells was reduced using U6 to inhibit JAK/STAT3 signal. Our findings reveal that enforced PEAK1 could activate JAK/STAT3 signal and promote EMT in melanoma cells.

## Conclusion

In this study, enforced PEAK1 expression induces EMT and promotes cell growth and metastasis *in vitro* and *in vivo* in melanoma cells through activating JAK/STAT3 signaling. Furthermore, targeting PEAK1 significantly decreases EMT and metastasis in melanoma cells through inhibiting JAK/STAT3 signaling. Therefore, targeting PEAK1 might be an effective therapeutic strategy for patients with melanoma.

## Highlights

1. Targeting PEAK1 expression inhibits invasion and proliferation in melanoma cells *in vitro*, and vice versa *in vivo*;
2. Targeting PEAK1 expression inhibits tumorigenesis and metastasis in melanoma *in vitro*, and vice versa *in vivo*;
3. PEAK1 activates JAK/STAT3 signals and induces epithelial–mesenchymal transition (EMT) in melanoma cells;

## References

[1] Siegel RL, Miller KD, Jemal A. Cancer statistics, 2015. CA Cancer J Clin. 2015;65(1):5–29.2555941510.3322/caac.21254

[2] Boire A, Brastianos PK, Garzia L, et al. Brain metastasis. Nat Rev Cancer. 2020;20(1):4–11.3178078410.1038/s41568-019-0220-y

[3] Korn EL, Liu PY, Lee SJ, et al. Meta-analysis of phase II cooperative group trials in metastatic stage IV melanoma to determine progression-free and overall survival benchmarks for future phase II trials. J Clin Oncol. 2008;26(4):527–534.1823511310.1200/JCO.2007.12.7837

[4] Eggermont AM, Spatz A, Robert C. Cutaneous melanoma. Lancet. 2014;383(9919):816–827.2405442410.1016/S0140-6736(13)60802-8

[5] Luís R, Brito C. Pojo M.Melanoma metabolism: cell survival and resistance to therapy. Adv Exp Med Biol. 2020;1219:203–223.3213070110.1007/978-3-030-34025-4_11

[6] Strickley JD, Jenson AB, Jung JY. Cutaneous metastasis. Hematol Oncol Clin North Am. 2019;33(1):173–197.3049767410.1016/j.hoc.2018.08.008

[7] Haradwaj U, Kasembeli MM, Robinson P, et al. Targeting janus kinases and signal transducer and activator of transcription 3 to treat inflammation, fibrosis, and cancer: rationale, progress, and caution. Pharmacol Rev. 2020;72(2):486–526.3219823610.1124/pr.119.018440PMC7300325

[8] Johnson DE, O’Keefe RA, Grandis JR. Targeting the IL-6/JAK/STAT3 signalling axis in cancer. Nat Rev Clin Oncol. 2018;15(4):234–248.2940520110.1038/nrclinonc.2018.8PMC5858971

[9] Ding C, Tang W, Fan X, et al. Overexpression of PEAK1 contributes to epithelial-mesenchymal transition and tumor metastasis in lung cancer through modulating ERK1/2 and JAK2 signaling. Cell Death Dis. 2018;9(8):802.3003828710.1038/s41419-018-0817-1PMC6056550

[10] Tan HX, Cao ZB, He TT, et al. TGFβ1 is essential for MSCs-CAFs differentiation and promotes HCT116 cells migration and invasion via JAK/STAT3 signaling. Onco Targets Ther. 2019;12:5323–5334.3130870210.2147/OTT.S178618PMC6615717

[11] Liu L, Nam S, Tian Y. 6-Bromoindirubin-3ʹ-oxime inhibits JAK/STAT3 signaling and induces apoptosis of human melanoma cells. Cancer Res. 2011;71(11):3972–3979.2161011210.1158/0008-5472.CAN-10-3852PMC3107399

[12] Wang Y, Kelber JA, Tran Cao HS, et al. Pseudopodium-enriched atypical kinase 1 regulates the cytoskeleton and cancer progression. Proc Natl Acad Sci U S A. 2010;107(24):10920–10925.2053445110.1073/pnas.0914776107PMC2890752

[13] Kelber JA, Klemke RL. PEAK1, a novel kinase target in the fight against cancer. Oncotarget. 2010;1(3):219–223.2130105010.18632/oncotarget.128PMC3057678

[14] Huang L, Wen C, Yang X, et al. PEAK1, acting as a tumor promoter in colorectal cancer, is regulated by the EGFR/KRas signaling axis and miR-181d. Cell Death Dis. 2018;9(3):271.2944954410.1038/s41419-018-0320-8PMC5833579

[15] Agajanian M, Campeau A, Hoover M, et al. PEAK1 acts as a molecular switch to regulate context-dependent TGF-beta responses in breast cancer. PLoS One. 2015;10(8):e0135748.2626786310.1371/journal.pone.0135748PMC4533969

[16] Croucher DR, Hochgräfe F, Zhang L, et al. Involvement of Lyn and the atypical kinase SgK269/PEAK1 in a basal breast cancer signaling pathway. Cancer Res. 2013;73(6):1969–1980.2337833810.1158/0008-5472.CAN-12-1472

[17] Tactacan CM, Phua YW, Liu L, et al. The pseudokinase SgK223 promotes invasion of pancreatic ductal epithelial cells through JAK1/Stat3 signaling. Mol Cancer. 2015 Jul 29;14:139.2621563410.1186/s12943-015-0412-3PMC4517651

[18] Kelber JA, Reno T, Kaushal S, et al. KRas induces a Src/PEAK1/ErbB2 kinase amplification loop that drives metastatic growth and therapy resistance in pancreatic cancer. Cancer Res. 2012;72(10):2554–2564.2258927410.1158/0008-5472.CAN-11-3552PMC3366503

[19] Runa F, Adamian Y, Kelber JA. Ascending the PEAK1 toward targeting TGFβ during cancer progression: recent advances and future perspectives. Cancer Cell Microenviron. 2016;3(1):e1162.2939216310.14800/ccm.1162PMC5790177

[20] Fu JJ, Lin P, Lv XY, et al. Low molecular mass polypeptide-2 in human trophoblast: over-expression in hydatidiform moles and possible role in trophoblast cell invasion. Placenta. 2009;30(4):305–312.1921765810.1016/j.placenta.2009.01.005

[21] Zheng H, Kang Y. Multilayer control of the EMT master regulators. Oncogene. 2014;33:1755–1763.2360412310.1038/onc.2013.128

[22] Lamouille S, Xu J, Derynck R. Molecular mechanisms of epithelial-mesenchymal transition. Nat Rev Mol Cell Biol. 2014;15:178–196.2455684010.1038/nrm3758PMC4240281

[23] Teng Y, Ross JL, Cowell JK. The involvement of JAK-STAT3 in cell motility, invasion, and metastasis. JAKSTAT. 2014;3(1):e28086.2477892610.4161/jkst.28086PMC3995737

[24] Strnadel J, Choi S, Fujimura K, et al. eIF5A-PEAK1 signaling regulates YAP1/TAZ protein expression and pancreatic cancer cell growth. Cancer Res. 2017;77(8):1997–2007.2838154710.1158/0008-5472.CAN-16-2594PMC5392372

[25] Smith A, Teknos TN, Pan Q. Epithelial to mesenchymal transition in head and neck squamous cell carcinoma. Oral Oncol. 2013;49(4):287–292.2318239810.1016/j.oraloncology.2012.10.009PMC3586749

[26] Bai Y, Sha J, Kanno T. The role of carcinogenesis-related biomarkers in the wnt pathway and their effects on epithelial-mesenchymal transition (EMT) in oral squamous cell carcinoma. Cancers (Basel). 2020;12(3):229–234.10.3390/cancers12030555PMC713958932121061

[27] TMM R-F, Brisson BK, Durham AC, et al. Characteristics of the epithelial-mesenchymal transition in primary and paired metastatic canine mammary carcinomas. Vet Pathol. 2018;55(5):622–633.2978879710.1177/0300985818776054PMC7993492

[28] Serrano-Gomez SJ, Maziveyi M, Alahari SK. Regulation of epithelial-mesenchymal transition through epigenetic and post-translational modifications. Mol Cancer. 2016;15:18.2690573310.1186/s12943-016-0502-xPMC4765192

[29] Agajanian M, Runa F, Kelber JA. We recently reported that Identification of a PEAK1/ZEB1 signaling axis during TGFβ/fibronectin-induced EMT in breast cancer. Biochem Biophys Res Commun. 2015;465(3):606–612.2629794810.1016/j.bbrc.2015.08.071

[30] Gao Q, Liu Q, Chen H. Circular RNA hsa_circ_0000117 accelerates the proliferation and invasion of gastric cancer cells by regulating the microRNA-337-3p/signal transducer and activator of transcription 3 axis. Bioengineered. 2021;12(1):1381–1390.3389636510.1080/21655979.2021.1918992PMC8806281

[31] Cui N, Sun Q, Liu H, et al. Long non-coding RNA LINC00511 regulates the expression of microRNA-625-5p and activates signal transducers and activators of transcription 3 (STAT3) to accelerate the progression of gastric cancer. Bioengineered. 2021;12(1):2915–2927.10.1080/21655979.2021.1940611PMC880682134224294

[32] Jin W. Role of JAK/STAT3 signaling in the regulation of metastasis, the transition of cancer stem cells, and chemoresistance of cancer by epithelial-mesenchymal transition. Cells. 2020;15;9(1):217.10.3390/cells9010217PMC701705731952344

[33] Li R, Huang Y, Lin J. Distinct effects of general anesthetics on lung metastasis mediated by IL-6/JAK/STAT3 pathway in mouse models. Nat Commun. 2020;11(1):642.3200579910.1038/s41467-019-14065-6PMC6994546

[34] Gupta P, Sharma Y, Viswanathan P, et al. Cellular cytokine receptor signaling and ATM pathway intersections affect hepatic DNA repair. Cytokine. 2020;127:154946.3183758610.1016/j.cyto.2019.154946

[35] Tan Q, Liu Z, Li H, et al. Hormesis of mercuric chloride-human serum albumin adduct on N9 microglial cells via the ERK/MAPKs and JAK/STAT3 signaling pathways. Toxicology. 2018;408:62–69.2998184110.1016/j.tox.2018.07.001

[36] Liang Q, Ma D, Zhu X, et al. RING-finger protein 6 amplification activates JAK/ STAT3 pathway by modifying SHP-1 ubiquitylation and associates with poor outcome in colorectal cancer. Clin Cancer Res. 2018;24(6):1473–1485.2928823510.1158/1078-0432.CCR-17-2133

[37] Lee IO, Kim JH, Choi YJ, et al. Helicobacter pylori CagA phosphorylation status determines the gp130-activated SHP2/ERK and JAK/STAT signal transduction pathways in gastric epithelial cells. J Biol Chem. 2010;285(21):16042–16050.2034809110.1074/jbc.M110.111054PMC2871473

